# Jumping to Conclusions Style along the Continuum of Delusions: Delusion-Prone Individuals Are Not Hastier in Decision Making than Healthy Individuals

**DOI:** 10.1371/journal.pone.0121347

**Published:** 2015-03-20

**Authors:** Suzanne Ho-wai So, Nate Tsz-kit Kwok

**Affiliations:** Department of Psychology, The Chinese University of Hong Kong, Hong Kong SAR, China; Maastricht University Medical Centre, NETHERLANDS

## Abstract

Literature comparing ‘jumping to conclusions’ (JTC) between patients and healthy controls has demonstrated the importance of the reasoning bias in the development of delusions. When groups that vary along the entire delusional continuum are included, the relationship between JTC and delusionality is less clear. This study compared JTC and delusional dimensions between 28 patients with delusions, 35 delusion-prone individuals and 32 non-delusion-prone individuals. Delusion proneness was defined by an established threshold based on the Peters et al. Delusions Inventory. Two versions of the beads task (85:15 and 60:40) were used to measure JTC. As hypothesized, patients manifested hastier data gathering than the two non-clinical groups on both beads tasks. However, delusion-prone individuals did not manifest a hastier decision making style than non-delusion prone individuals. Instead, non-delusion-prone participants showed more JTC bias than delusion-prone individuals on the easier beads task. There was no evidence for a dose-response relationship between JTC and delusional dimensions, with correlations between JTC and PDI scores found in the non-delusion-prone group only. The present finding confirms the link between an extreme JTC bias and the presence of clinical delusions, and argues against a linear relationship between JTC and delusionality along the symptomatic continuum.

## Introduction

‘Jumping to conclusions’ (JTC) reasoning bias refers to a tendency to make decisions based on insufficient information in ambiguous situations [1]. Studies reported that JTC is found in 70% of individuals with delusions, and this hasty decision making style has been theorised as a predisposing factor for the development of delusions (see reviews in [2], [3], [4]). As evidence supporting the relationship between JTC and delusions accumulates, cognitive interventions have recently been developed to target this reasoning bias [5–6].

Large-scale population studies have consistently reported an overlap in psychotic symptoms between clinical and non-clinical groups [7–16]. These reports have led to a shift from the traditional categorical view to a continuum approach of understanding psychosis, where clinical delusions and non-delusional beliefs are suggested as two extreme ends of the same spectrum [7, 16–18]. This raises the following question: how does JTC, which is considered to predict the development of delusions, relate to delusionality along the symptomatic continuum?

Most investigations of JTC and delusionality either compared patients with non-clinical controls, or compared non-clinical individuals with high vs. low delusion-proneness (see review by [4]). As reviewed by Garety and Freeman [4], non-clinical studies of JTC yielded mixed evidence, with some studies reporting hastier decision-making in individuals with high compared to low delusion-proneness (e.g. [19–21]), whereas others reported no significant group difference [22–24].

A potentially more robust design to investigate the link between JTC and delusionality would be studies that encompass the full symptomatic continuum, comparing patients, individuals with high delusion proneness and individuals with low delusion proneness. This design allows for (i) comparison of JTC bias across clinical and non-clinical groups varying on delusionality, and (ii) investigation of dose-response relationship between JTC and severity of delusions across groups. To date, four studies took this approach [25–28].

Despite comparable patient symptom profiles across studies, the group comparison results were divergent. Van Dael et al. [27] reported a graded difference in JTC across groups, with the highest proportion of patients giving a definite rating after seeing only one bead on the beads task, followed by the delusion-prone group and then the non-delusion-prone group. Van Dael et al. [27] also found that the association between level of psychosis liability and JTC was stronger in individuals with delusions than those without, suggesting a dose-response relationship between JTC and delusions. Although a similar trend of graded JTC pattern across groups was observed by Balzan et al. [25], the difference in JTC (defined by definite certainty rating on the first bead) between the two non-clinical groups did not reach statistical significance. On the contrary, Freeman et al. [26] and Warman et al. [28] found that JTC was unique to the clinical group and not associated with delusions in the non-clinical groups. In both studies, the delusion-prone individuals actually gathered more information than the non-delusion-prone individuals. According to Warman et al. [28], the clinical group gave the most definite decisions after two beads, followed by the non-delusion-prone and then the delusion-prone group. In both Freeman et al. [26] and Warman et al. [28], the difference between the two non-clinical groups was not significant.

Warman et al. [28] proposed a possible explanation for their finding of a lack of stepped difference in JTC—that delusion-prone individuals substantially adjust their data gathering strategies to a difficult task. Both Freeman et al. [26] and Warman et al. [28] used the 60:40 version of the beads task only, whereas Balzan et al. [25] and Van Dael et al. [27] used an easier version (with a 90:10 or 85:15 ratio of bead colours respectively). It is unclear to what extent the lack of stepped difference along the continuum in Freeman et al. [26] and Warman et al. [28] was related to the more ambiguous beads task used.

Apart from variations in the JTC task, the above studies also differed in their criteria for delusion-proneness, which might also contribute to the divergent findings as illustrated. Van Dael et al. [27] used the Community Assessment of Psychic Experiences scale positive dimension [29], whereas Freeman et al. [26] used the Paranoid Thought Scale [30]. Compared to these two scales, the Peters et al. Delusions Inventory (PDI) [31] was more widely applied to measure delusion proneness [19, 21–25, 28]. Both Balzan et al. [25] and Warman et al. [28] determined delusion-proneness based on median split of the PDI total score. The PDI total score is an aggregate score of the number of delusion-like beliefs endorsed on the PDI and three dimensions of delusions (conviction, distress and preoccupation). Therefore, an individual who endorses only a few highly distressing or preoccupying beliefs may have a similar PDI total score with an individual who endorses many non-distressing or non-preoccupying beliefs. Instead of the total score, Preti et al. [32] reported a reliable cutoff criterion using number of beliefs on the PDI. According to Preti et al. [32], a threshold of eight delusion-like beliefs on the PDI reliably discriminated patients with psychosis from healthy individuals, with 74% sensitivity and 79% specificity. With the expected high negative predictive value of 96%, Preti et al. [32] recommended PDI as a tool for assessing psychosis proneness among non-clinical samples.

The present study aimed to expand on the existing literature and revisit the tendency of JTC varying along the delusional spectrum using both the easier (85:15) and harder (60:40) versions of the beads task, across groups that are defined by a reliable psychometric cutoff criterion.

Based on previous studies, key hypotheses were as follows:

1. on the easier (85:15) beads task, the number of beads drawn to decision will be the smallest in the clinical group, followed by the delusion-prone group, and then the non-delusion-prone group;
2. on the harder (60:40) beads task, the number of beads drawn to decision will be the smallest in the clinical group, followed by the delusion-prone group, and then the non-delusion-prone group;
3. there will be a stronger association between data gathering and PDI scores in the clinical group than the non-clinical groups.

## Methods

This study was approved by the New Territories West Cluster Research Ethics Committee (Reference number: NTWC/CREC/476/06), Hong Kong.

### Participants

Patients were recruited from an early intervention programme at Castle Peak Hospital for psychosis in Hong Kong. Adult patients with a casenote diagnosis of schizophrenia spectrum disorder with present delusions were included. Exclusion criteria were learning disability, organic brain disorders and drug-induced psychosis. Before patients were invited to take part in the study, their capacity to give consent to study participation was ascertained by their treating psychiatrists. Non-clinical controls were recruited from educational and community institutes. Only adults with no personal or family history of psychiatric illness were included in the study. All participants gave written informed consent to join the study in person.

### Measures

#### Positive and Negative Syndrome Scale (PANSS) [33]

Symptomatology of patients was assessed by their treating psychiatrists using PANSS. PANSS consists of symptoms commonly reported in schizophrenia, grouped into three subscales: positive (7 items), negative (7 items), general psychopathology (16 items), and a total score. Good psychometric properties of PANSS have been reported [33].

#### Beads Tasks

‘Jumping to conclusions’ (JTC) was assessed using the 85:15 and 60:40 versions of the beads task [34–35]. All participants completed the 85:15 task first, followed by the 60:40 task. In the 85:15 beads task, two jars containing orange and black beads in respective ratios of 85:15 and 15:85 are presented on a laptop computer. Beads are drawn according to a predetermined order unknown to the participant, one by one with replacement. Upon presentation of each bead, the participant can either make a decision on which jar the beads are drawn from or request to view more beads. All the beads that have been drawn remain in view. The procedure of the 60:40 beads task is the same as the 85:15 version, but the two jars contain blue and red beads in a ratio of 60:40 and 40:60 respectively [36]. The predetermined sequences of bead presentation in the two tasks (as shown below) are similar to previous studies using the same tasks [34–38]:

85:15 beads task (○ = orange, ● = black):
○ ○ ○ ● ○ ○ ○ ● ○ ○ ○ ● ○ ○ ● ○ ○ ○ ○ ○
60:40 beads task (○ = blue, ● = red):
○ ● ● ○ ○ ● ○ ○ ○ ● ○ ○ ○ ○ ● ● ○ ● ● ○

The number of draws to decision (DTD) was recorded as a measure of data-gathering style. Garety et al [39] suggested dichotomizing the DTD measure into presence and absence of an extreme JTC bias, with two beads or fewer classified as an extreme JTC response, and this method of assessing JTC has been used in numerous studies (e.g. [35, 39–42]).

#### The 21-item Peters et al. Delusions Inventory (PDI-21) [31]

PDI-21 [31] is a self-rated questionnaire of delusional ideation. Participants were asked if they had experienced any of the 21 delusion-like beliefs (yes/no), and for each endorsed belief, to rate their degrees of conviction, distress and preoccupation on a 5-point Likert scale respectively. In the original PDI-21, the conviction score, distress score, and preoccupation score are obtained by adding up the dimension ratings for all the endorsed beliefs (range 0–105 for each dimension). The PDI total score is the sum of all the dimension scores and the number of beliefs (range 0–336). In order to examine the relationship between reasoning bias and delusional dimensions more specifically (independent of the number of beliefs endorsed), we included in this study all the original PDI measures as well as average levels of conviction, distress, and preoccupation (range 0–5 for each dimension). This strategy of analysing average dimension scores has been adopted in recent PDI studies [32, 43].

All participants completed the PDI and the beads tasks in the presence of the researcher.

### Statistical analysis

To compare JTC style across the three groups (clinical, delusion-prone, and non-delusion-prone groups), group difference in DTD was tested using one-way ANOVAs, whereas prevalence of JTC bias and error rates were compared using chi-square tests (or Fisher’s exact tests in case of any expected value smaller than 5). Where group differences were found, these were followed by Bonferroni pairwise comparisons (for continuous variables) and 2x2 chi-square or Fisher’s exact tests (for categorical variables). To explore the relationship between beads task performance and PDI dimensions, a series of regression analyses with the PDI scores as IVs and various beads task measures as DVs were performed using data from the three groups respectively.

## Results

### Demographics and delusional dimensions across groups

This sample (N = 95) consisted of 28 patients with delusions and 67 individuals from the community. Among the non-clinical participants, the mean number of PDI beliefs endorsed was 7.54 (SD = 3.20, median = 8, range = 1–14), whereas mean PDI total score was 66.5 (SD = 33.15, median = 65, range = 4–132). According to Preti et al (2007), 35 (52.2%) individuals endorsed eight or more delusion-like experiences on the PDI and were categorised into the ‘delusion-prone’ group, whereas the remaining 32 (47.8%) were categorised into the ‘non-delusion-prone’ group. Preti et al’s (2007) cut-off of eight PDI beliefs coincides with the median number of beliefs endorsed in this sample. Therefore, median split of PDI number of beliefs would yield the same grouping of non-clinical individuals as Preti et al’s (2007) psychometric cutoff.

Gender distribution was comparable across groups (Percentage of male participants: 46.4% in clinical group, 40.0% in delusion-prone group, 28.1% in non-delusion-prone group; χ^2^(2, n = 95) = 2.23, *p* = .328). There was a significant group difference in age (F(2,92) = 3.29, *p* = .042), with a non-significant trend of the patients (mean 21.25 years; SD = 3.65) being older than the delusion-prone group (mean 19.51 years; SD = 2.37; *p* = .058). Year of education differed across groups (F(2,88) = 18.52, *p* <. 001), with patients having less education (mean 10.88 years; SD = 2.59) than both the delusion-prone (mean 13.60 years; SD = 1.63; *p* <. 001) and the non-delusion-prone (mean 13.84 years; SD = 1.76; *p* <. 001) groups.

Information on medication was available for 26 patients. Fourteen patients were on atypical antipsychotics (Risperidone, Olanzapine, Quetiapine, Amisulpiride, Clozapine and Ziprasidone), nine were on typicals (Zuclopenthixol, Haloperidol, and Flupentixol), and three were not on any anti-psychotics. The mean dose of antipsychotics in chlorpromazine equivalents [44–45] was 244.32 mg/day (SD = 170.44).

In the clinical group, the average PANSS scores were as follows: positive 19.50 (SD = 6.94, range 8–33), negative 16.79 (SD = 6.53, range 7–28), general psychopathology 37.25 (SD = 13.12, range 16–57), and delusion item score 3.71 (SD = 1.24, range 2–5).

PDI scores of the groups are presented in Table 1. There was a significant group difference in PDI total score (*p* <. 001) and number of delusion-like beliefs endorsed (*p* <. 001). Post-hoc Bonferroni tests revealed a significantly higher PDI total score in the delusion-prone group than patients (*p* <. 001), and a significantly higher PDI total score in patients than the non-delusion-prone group (*p* = .001). A similar graded pattern was found in the number of delusion-like beliefs endorsed, with the delusion-prone group endorsing significantly more delusion-like beliefs than patients (*p* <. 001), and patients endorsing more beliefs than the non-delusion-prone group (*p* = .003).

**Table 1:** Mean (SD) of the Peters et al. Delusions Inventory (PDI) scores.

	Patients	Delusion-Prone	Non-delusion-prone	Group difference*
PDI Total score	(n = 26)	(n = 34)	(n = 32)	F(2,89) = 25.619
	69.38(40.50)	90.68(22.65)	40.81(20.89)	*p*<.001
Number of beliefs	(n = 28)	(n = 35)	(n = 32)	
	7.11(3.82)	10.00(1.80)	4.84(1.97)	F(2,92) = 32.985
	range:1–14	range:8–14	range:1–7	*p*<.001
PDI Conviction	(n = 26)	(n = 34)	(n = 32)	
Total	21.38(12.18)	30.32(8.80)	13.91(6.86)	F(2,89) = 1.015
Per belief	2.81(0.87)	3.02(0.63)	2.77(0.80)	*p* = .367
PDI Distress	(n = 26)	(n = 35)	(n = 32)	
Total	20.62(13.12)	24.83(7.38)	10.81(6.64)	F(2,90) = 5.197
Per belief	2.70(0.87)	2.48(0.59)	2.09(0.75)	*p* = .007
PDI Preoccupation	(n = 27)	(n = 35)	(n = 32)	
Total	19.19(13.45)	25.37(7.00)	11.25(6.46)	F(2,91) = 2.637
Per belief	2.49(0.81)	2.53(0.53)	2.17(0.72)	*p* = .077

*Group differences of delusional dimensions pertain to the ‘per belief’ scores

For delusional dimensions, significance of group difference was tested for average level of dimensions per belief, and not for total dimension scores. There was a significant group difference in delusional distress, with the non-delusion-prone group lower than the clinical group (*p* = .007). Group difference was not significant for delusional preoccupation and conviction (*p* >. 05).

### Data-gathering style across groups

Performance of the two versions of the beads task across groups is presented in Fig. 1, Tables 2 and 3. Across groups, number of beads drawn to decision was significantly lower in the easier beads task (85:15 task) than the more difficult one (60:40 task): patients (mean difference = -0.57; SD = 1.48; *p* = .05), delusion-prone individuals (mean difference = -4.06; SD = 3.02; *p* <. 001) and non-delusion-prone individuals (mean difference = -2.72; SD = 2.75; *p* <. 001). Age was not significantly correlated with the number of draws to decision (DTD) in any of the groups for either beads task (*p* >. 05). Level of education, however, was correlated with DTD on the 60:40 beads task within the delusion-prone group only (r = .39, *p* = .019). Level of education was not correlated with DTD on the 85:15 beads task in any group, or with prevalence of JTC bias and error rate on the 60:40 task in any group (*p* >. 05).

**Fig 1:** Performance of the two beads tasks across groups.

**Table 2:** Performance on the 85:15 beads task across groups.

	Patients (N = 28)	Delusion-Prone (N = 35)	Non-delusion-prone (N = 32)	Group difference
Draws to decision	1.75(2.46)	5.20(3.97)	4.03(4.08)	F(2,92) = 7.112
	range:1–14	range:1–17	range:1–20	*p* = .001
JTC bias^a^(DTD≦2)	92.9%	20.0%	53.1%	χ^2^(2,n = 95) = 33.125
				*p*<.001
JTC bias^b^ (DTD = 1)	71.4%	8.6%	28.1%	χ^2^(2,n = 95) = 28.181
				*p*<.001
Error rate	21.4%	2.9%	9.4%	*p* = .0688
				FET two tailed

^a^Defined by making a decision after viewing two or fewer beads

^b^Defined by making a decision after viewing one bead only

**Table 3:** Performance on the 60:40 beads task across groups.

	Patients (N = 28)	Delusion-Prone (N = 35)	Non-delusion-prone (N = 32)	Group difference
Draws to decision	2.32(3.65)	9.26(4.52)	6.75(5.36)	F(2,92) = 17.847
	range:1–20	range:1–20	range:1–20	*p*<.001
JTC bias^a^(DTD≦2)	78.6%	8.6%	25.0%	χ^2^(2,n = 95) = 35.640
				*p*<.001
JTC bias^b^ (DTD = 1)	64.3%	8.6%	18.8%	χ^2^(2,n = 95) = 25.954
				*p*<.001
Error rate	39.3%	5.7%	21.9%	χ^2^(2,n = 95) = 10.568
				*p* = .005

^a^Defined by making a decision after viewing two or fewer beads

^b^Defined by making a decision after viewing one bead only

#### Hypothesis 1: on the easier (85:15) beads task, the number of beads drawn to decision will be the smallest in the clinical group, followed by the delusion-prone group, and then the non-delusion-prone group

As shown in Table 2, there was a significant group difference in DTD on the 85:15 beads task (*p* = .001). Post-hoc Bonferroni tests showed that patients drew significantly fewer beads than the delusion-prone group (*p* = .001). There was a statistical trend that patients drew fewer beads than non-delusion-prone individuals (*p* = .052), whereas the two non-clinical groups did not differ from each other (*p* = .576).

With a three-by-two chi-square test, a significant group difference in prevalence of JTC bias (defined by decision after viewing two or fewer beads) was found across all groups (χ^2^(2, n = 95) = 33.125, *p* <. 001). Two-by-two chi-square tests revealed that JTC was more prevalent in patients than in the non-delusion-prone group (χ^2^(1, n = 60) = 11.61, *p* = .001), and more prevalent in the non-delusion-prone group than in the delusion-prone group (χ^2^(1, n = 67) = 7.979, *p* = .005).

Extreme JTC bias (defined by decision after viewing one bead only) was also significantly different across the three groups (χ^2^(2, n = 95) = 28.181, *p* <. 001). Two-by-two chi-square tests revealed that an extreme JTC bias was more common in patients than in non-delusion-prone group (χ^2^(1, n = 60) = 11.214, *p* = .001), and more common in the non-delusion-prone group than in the delusion-prone group (χ^2^(1, n = 67) = 4.347, *p* = .037).

A three-by-two Fisher’s exact test revealed no significant group difference in error rate (*p* = .0688, two tailed).

#### Hypothesis 2: on the harder (60:40) beads task, the number of beads drawn to decision will be the smallest in the clinical group, followed by the delusion-prone group, and then the non-delusion-prone group

As shown in Table 3, there was a significant group difference in DTD on the 60:40 beads task (*p* <. 001). Post-hoc Bonferroni tests showed that DTD was significantly fewer in patients than in both delusion-prone (*p* <. 001) and non-delusion-prone (*p* = .001) groups, which did not differ from one another (*p* = .085).

A three-by-two chi-square test revealed a significant group difference in prevalence of JTC (defined by decision after viewing two or fewer beads) (χ^2^(2, n = 95) = 35.64, *p* <. 001). Two-by-two chi-square tests showed that JTC was more common in the clinical group than both the delusion-prone (χ^2^(1, n = 63) = 31.845, *p* <. 001) and non-delusion-prone (χ^2^(1, n = 60) = 17.143, *p* <. 001) groups, which did not differ from one another (*p* = .070).

Extreme JTC (defined by decision after viewing one bead only) was different across groups (χ^2^(2, n = 95) = 25.95, *p* <. 001). Two-by-two chi-square tests showed a higher prevalence of extreme JTC bias in patients relative to both delusion-prone (χ^2^(1, n = 63) = 21.729, *p* <. 001) and non-delusion-prone (χ^2^(1, n = 60) = 12.902, *p* <. 001) groups. The two non-clinical groups did not differ from one another (*p* = .292, Fisher’s exact test two-tailed).

There was a significant group difference in error rate (χ^2^(2, n = 95) = 10.568, *p* = .005). Two-by-two chi-square tests revealed significant group difference in error rate between patients and the delusion-prone group (χ^2^(1, n = 63) = 10.705, *p* = .001) only.

#### Hypothesis 3: There will be a stronger association between data gathering and PDI scores in the clinical group than the non-clinical groups

For the clinical and the delusion-prone groups, linear regression analyses of PDI scores as IVs and beads task measures as DVs failed to generate any statistically significant model (*p* >. 05). Delusional dimensions on the PDI did not predict any of the beads task measures.

For the non-delusion-prone group, the PDI total score significantly predicted DTD on the 85:15 task (Beta = 0.499, SE = 0.031, *t* = 3.156, *p* = .004), and delusional preoccupation significantly predicted DTD on the 60:40 task (Beta = 0.471, SE = 1.197, *t* = 2.923, *p* = .007). Delusional preoccupation also significantly predicted JTC bias of the 60:40 task (B = -3.938, SE = 1.902, Wald χ^2^ (1) = 4.288, *p* = .038).

## Discussion

This study compared the beads task performance in patients with delusions, participants from the community who met the criterion of delusion proneness, and non-delusion-prone individuals. We found that, on the less ambiguous version of the beads task (with the colour ratio 85:15), the jumping to conclusions (JTC) bias was stronger in patients, followed by non-delusion-prone individuals, and then delusion-prone individuals. On the more ambiguous version of the beads task (with an 60:40 colour ratio), the pattern of group difference was the same but the difference between the two non-clinical groups was not statistically significant. A hasty decision making style was more prevalent among patients than the non-clinical groups on both versions of the beads task.

With the same pattern of group difference for both beads tasks in our study, Warman et al.’s [28] hypothesis that delusion-prone individuals, in particular, adjusted their data gathering strategies to a difficult task was not supported. On the contrary, consistent with other studies that included both versions of the beads task (e.g. [36, 38, 40]), all groups drew significantly more beads in the more difficult version. This suggests that clinical and non-clinical participants, across studies, understand and respond to the varying task instructions and demands.

The finding that patients had a more hasty decision-making style than non-clinical participants replicated previous studies (e.g., [2, 4, 37, 41]), confirming the role of JTC in predicting the presence of delusions. However, the hypothesised stepped decrease in JTC bias along the delusional continuum (i.e. patients > delusion-prone group > non-delusion-prone group), especially the expected difference between the two non-clinical groups, was not found. On both beads tasks, the delusion-prone individuals actually gathered more information to make decisions than the non-delusion-prone individuals, which replicated findings in Freeman et al. [26] and Warman et al. [28]. Despite the different ways delusion-proneness was measured, the DTD and prevalence of JTC bias of the non-clinical groups reported in the present study were comparable to both said studies. However, the difference between the non-clinical groups (i.e. a stronger JTC bias in non-delusion-prone than delusion-prone individuals) reached statistical significance for the first time in the present study. With at least three published studies to date reporting less JTC in delusion-prone than non-delusion-prone individuals, it is conceivable that the predictive nature of JTC on delusions may not be linear.

Evidence supporting the role of JTC in delusion development is most marked when patients are compared with non-clinical individuals (see review by [4]). When at-risk or delusion-prone groups are included, the effect of JTC on delusions becomes less explicit. This may simply be due to the smaller difference in both JTC tendency and delusion severity across comparison groups. For example, non-clinical studies that reported more JTC in delusion-prone than non-delusion-prone individuals tended to adopt a percentile split, yielding two non-clinical groups more widely apart on delusion-proneness than studies using a median split [19, 21]. However, studies that investigated the link between JTC and delusion-proneness based on median split grouping or correlation approaches did not provide consistent results [20, 22, 23, 25, 28, 46].

Another possibility is that the JTC style only reliably distinguishes risk of delusions when it becomes extreme (i.e. decision after viewing only 1 to 2 beads, as in the clinical group). After the first few bead draws, the subsequent beads requested may have a diminishing marginal effect in differentiating risk of delusions. In fact, with studies including clinical samples only, the systematic association between JTC and severity of delusions is not consistently reported (e.g. [47–48]). Similarly, clinical and non-clinical studies using multi-dimensional measures found inconsistent results regarding the association between JTC and dimensions of delusions [22, 23, 49]. We did not find a closer link between JTC and delusional ideation in the clinical group as compared with healthy controls. Therefore, while the JTC bias is associated categorically with the presence of delusions, there is less evidence supporting a linear relationship between JTC and severity of or predisposition to delusions. As suggested by Van Dael et al. [27], it is possible that cognitive processes in patients with delusions are not dysfunctional under optimal environmental conditions, but are more susceptible to impact from adverse events than those of individuals who never have delusional experiences. Bentall et al. [50] argued for a combination of affective and cognitive processes (including JTC) in contributing to paranoia across clinical and non-clinical groups. Therefore, a more reliable prediction of the risk of developing delusions may take into account other psychosocial factors that may mediate or interact with JTC.

Using an established PDI threshold [32], the present study included delusion-prone individuals who reported delusional ideation that was not less prominent than the clinical group. Rather, delusion-prone individuals in this study endorsed a greater number of delusion-like beliefs and had a higher PDI total score than patients. Previous studies using the PDI have reported number of beliefs endorsed in non-clinical individuals ranging from 5.40 to 11.32 [23, 51–54]. Mean number of PDI beliefs endorsed in the present study (7.54) posits our non-clinical sample within the wide range of previous studies. On the other hand, mean number of beliefs endorsed by our patients (7.11) appeared to be smaller than that reported by previous studies (e.g. 11.8 in Peters et al. [55], 8.76 in Lim et al. [52]). The mean PDI total score in our patients (69.38) was also smaller than in previous studies (e.g. 128.14 in Kao et al. [51]; 91.04 in Lim et al. [52]). It is possible that our patients, who had first-episode psychosis, had lower delusional ideation than patients in other studies. However, given that PDI was designed to assess a set number of standard delusional ideation (or delusion-like or unusual beliefs), patients who score high on a clinical rating scale of delusions do not necessarily endorse many beliefs on the PDI. Despite the level of PDI total score and number of beliefs in the delusion-prone group, delusional distress was significantly higher in patients than in non-delusion-prone individuals, which replicates previous findings and confirms the importance of delusional distress in differentiating clinical and non-clinical populations [54, 56]. Altogether, the present findings make one wonder how the delusion-prone individuals, with a high level of delusional ideation but a lack of a hasty decision-making style, maintain their functioning without the need for clinical care. It has been postulated that JTC and belief flexibility may jointly contribute to delusion development, where a lack of JTC creates doubt for the individual to consider alternative explanations [26, 39, 54]. This theory has been tested in clinical samples only [39, 57].

The present study has several limitations. Data-gathering style was measured using number of beads drawn to decision, which was suggested to be the most reliable measure of JTC in differentiating individuals with and without delusions [2]. However, we did not record participants' confidence of their decision, which had anecdotally been reported as different between groups varying in delusion-proneness [28]. Moreover, patients were recruited based on casenote diagnoses. Although present delusion was checked using the PANSS, a standardized diagnostic procedure would increase assessment reliability. This study also lacked a formal screening procedure to confirm the absence of mental illness in the non-clinical individuals. In addition, our patients were not matched with the non-clinical individuals on age and year of education. Although our major findings were not affected by this difference, a perfectly matched control group would strengthen the interpretability of the results. It will also be beneficial to have a measure of general intelligence, which has been associated with JTC bias in some studies [23, 27, 37].

Future research on JTC, using multiple measures, as well as its interaction with belief flexibility in delusion-proneness may extend our understanding of the role of cognitive processes between the non-clinical and clinical ends of the delusion spectrum. This can then be followed by examining the effect of interventions targeting specific cognitive processes in reducing sub-clinical delusions or in delaying transition into psychosis (e.g. metacognitive training) [5–6].
